The article "Birthweight predicts glomerular filtration rate in adult-life: population based cross sectional study" was retracted in 2022. Reasons: no approval from a third party; copyright claims.

# Birthweight predicts glomerular filtration rate in adult-life: population based cross sectional study

**DOI:** 10.1080/0886022X.2021.1915798

**Published:** 2021-04-26

**Authors:** Issa Al Salmi, Suad Hannawi

**Affiliations:** a The Medicine Department, The Royal Hospital, Muscat, Oman; b The Medicine Department, MOHAP, Dubai, UAE

**Keywords:** Birth weight (BW), low birth weight (LBW), intra-uterine growth retardation (IUGR), non-communicable diseases (NCD), estimated glomerular filtration rate (eGFR), albumin creatine ratio (ACR)

## Abstract

**Introduction:**

Worldwide, there is a global progressive rise of chronic kidney disease. In parallel, children born after intra-uterine growth retardation are surviving to adult-life and beyond. This study describes the association of birthweight with and estimated glomerular filtration rate (eGFR).

**Methods:**

Australian Diabetes, Obesity and Lifestyle (AusDiab) study participants were asked to complete a birthweight questionnaire. The associations between birthweight and eGFR were determined.

**Results:**

A total of 4502 reported information related to their birthweight, with the other responders did not provide a value. The birthweight of the participants ranged from 0.4 to 7.0 kg with a mean-(SD) of 3.37 (0.7) kg. The mean (95%CI) birthweight was lower for females, 3.28 (0.6) kg, when compared to males, 3.5 (0.7) kg. Eight percent had a birthweight less than 2.5 kg. The eGFR was strongly and positively associated with birthweight, with people in the lowest sex-specific birthweight-quintiles having the lowest mean eGFR. This relationship persisted with adjustment for confounding factors. The OR(CI) for eGFR <10th-percentile (<61.4 ml/min for females and <73.4 for males) for people in the lowest vs. the higher birthweight-quintile was 2.19 (95%CI 1.14–4.2) for females and 2.37 (1.1–5.3) for males, after adjustment for other factors.

**Conclusions:**

Birthweight had a positive relationship with eGFR. Possible explanations include an association of birthweight with nephron-endowment. From a global health perspective but more in developing countries and in populations in epidemiologic transition, where substantially lower birthweights coexist with recently improved infant and adult survivals, the overall impact of this phenomenon on the population health profile could be more substantial.

## Introduction

The tsunami of non-communicable diseases (NCD) had spread throughout the globe. Similarly, chronic kidney disease is rising worldwide. Also, the survival of babies with intra-uterine growth retardation to adult life has improved over the last few decades. In recent years, there has been great interest in the relationship of fetal development to diseases in later life [1–5]. Developmental origins of health and disease (DOHaD), Barker's hypothesis, originates from epidemiological studies of birth and mortality records which showed an association between infant mortality rates and later adult deaths. It, also, found a correlation between birthweight and mortality rates of adult from ischemic heart disease [6]. Barker hypothesis had set up the groundwork for a broad range of knowledge and understanding of the prenatal and perinatal origin of non-communicable diseases [7–9]. Dietary deficiencies and various other insults or lesions are accountable for stress during pregnancy that occur during the perinatal critical period [10,11]. These insults produce an effect through the programming of various hormonal responses and that programming takes place through epigenetic changes. Human beings could easily cope with an environment of limited dietary resources [12,13]. However, when born in an environment of nutritional abundance, which is compounded with a sedentary lifestyle, disease programming directs them to various metabolic disorders. Knowing that programming takes place through epigenetic changes, these mechanisms have transgenerational consequences as the result of interaction between genetic programming and an adverse environment [14].

The article "Birthweight predicts glomerular filtration rate in adult-life: population based cross sectional study" was retracted in 2022. Reasons: no approval from a third party; copyright claims.

Low birthweight is the widely used surrogate marker of adverse events that happened in prenatal life *in utero*. In recent times, low birth weight has been suggested that people with low birthweights are inclined to higher risk for development of various non communicable disease than those with normal birthweights. These diseases, which may include risk factors for various metabolic and cardiovascular diseases such as obesity, diabetes, hypertension, lipids abnormalities and various other metabolic disorders.

The mechanism of association between adult chronic kidney disease (CKD) and birth weight association are still elusive. Because various kidney dysfunction abnormalities are a strong risk factor for end-stage kidney disease (ESKD), many researchers have tried to clarify the relationship between birth weight and these abnormalities. These studies, however, were performed in selected populations, based on geographical location, ethnicity, and/or professional status. None have looked at the phenomenon in a general adult population.

The relationship of birthweight to the risk factors of chronic diseases in adult life, what being called the fetal origin of disease, had being critiqued for number of reasons. These reasons include that researchers had obtained significant results after adjusting for body size and or that various lifestyle including physical activity, smoking status, alcohol intake, family history and socioeconomic status have not addressed in the assessment of these relationship [15–18]. In addition, females and males differ in their birthweight throughout all populations across the world and as such the relationship between birthweight and adult disease requires separate assessment for females and males. The relationships of birthweight and estimated glomerular filtration rate (eGFR) in the general adult population have not been addressed. Any positive relationship between birthweight and eGFR could provide a predictor for future kidney disease.

The article "Birthweight predicts glomerular filtration rate in adult-life: population based cross sectional study" was retracted in 2022. Reasons: no approval from a third party; copyright claims.

Hence, this study aimed to evaluate the relationship between birthweight and components of kidney function including urinary albumin-creatinine ratio (ACR), serum creatinine (SCr) and with the eGFR.

## Methods

### Participants

The AusDiab study is a national, population-based, longitudinal study in which participants were recruited from a stratified sample of Australians aged ≥ 25 years, residing in 42 randomly selected urban and non-urban areas (Census Collector Districts) of the six states of Australia and the Northern Territory [19]. The study was approved by the International Diabetes Institute ethics committee (Melbourne, Australia). Written informed consent was obtained from all individuals.

### Measurements

The AusDiab Birth weight cohort examines the relationship between birthweight and development of chronic diseases in adult life. The methods of the AusDiab study had been discussed in detail previously [19]. The consented participants were asked to present at a local screening venue and completed a series of various questionnaires, physical examinations, and specific laboratory tests such as metabolic status, various cardiac risk factors, and kidney parameters. In addition, questionnaires were completed during interviews to assess various lifestyles issues and habits which include smoking status, alcohol consumption, leisure-time physical activity and television viewing. Assessment of socioeconomic status was based on education [20], income [20] and dwelling type (house owner vs. non house owner).

Various questions about birthweight were included in the follow-up 2005-AusDiab study. Participating consenting individuals were asked to declare their birthweight, how accurate is their stated birthweight and from where their stated birthweight was obtained. The birth weight data were linked to the various kidney tests and parameters of the AusDiab survey study. Participating individuals were divvied into gender-specific quintiles of birthweight for further statistical analysis. Also, birth weight was divided as normal birthweight if it is 2.5 kg or above, and as low birthweight if < 2.5 g as dichotomous variable.

The article "Birthweight predicts glomerular filtration rate in adult-life: population based cross sectional study" was retracted in 2022. Reasons: no approval from a third party; copyright claims.

Apart from those who were (i) chairbound, (ii) pregnant or (iii) too unsteady on their feet, all participating consented individuals underwent anthropometric measurements while wearing light clothing and no footwear during the initial encounters of conduction of the study. The height was assessed to the nearest 0.5 cm using a stadiometer, and weight was quantified using a mechanical beam balance, and was noted to the nearest 0.1 kg. The body mass index was determined as weight (kg)/height (m)^2^, and was defined as < 25 kg/m^2^ and ≥ 25 kg/m^2^ according to World Health Organization criteria [21].

Blood was collected by venipuncture after an overnight fast of at least 10 h. Blood specimens collected were centrifuged on-site and transported daily with urine samples to the central laboratory. SCr was measured by the modified kinetic Jaffe reaction using the Olympus AU600 auto-analyzer and the coefficient of variation was <1.9%. Urinary albumin and creatinine levels were determined in a spot morning urine specimen by means of enzymatic methods (Olympus AU600 analyzer).

The AusDiab study is a longitudinal population-based study examining the natural history of diabetes and pre-diabetes. As the participants are not a population with chronic kidney disease, GFR was estimated using the Cockcroft Gault (CG) equation [22]. The estimated GFR was obtained using the CG method the formula as follows [22], estimated GFR = ((140- age × weight)/(0.81 × SCr in µmol/l)) × 0.85 if female. This method is considered the more accurate one to apply in healthy subjects with normal GFR values [23]. CG estimates have been found to correlate well with gold-standard measures of GFR in studies examining a similar range of subjects to those studied in AusDiab, including those with type 2 diabetes mellitus, the obese, and the ambulatory elderly [24]. Although indexing GFR to body surface area (BSA) is controversial [25], we also describe GFR estimates adjusted for BSA, using the formula: weight^(0.425)^ × height^(0.725)^ × 0.20247 m^2^ [26].

### Statistical analysis

The Student’s *t*-test was used to compare differences in mean values of baseline characteristics among (i) responders and non-responders and (ii) those classified as having LBW (<2.5 kg) and those classified as having normal birthweight (≥2.5 kg). Albuminuria, urinary creatinine and ACR were not normally distributed and were logarithmically transformed. The other continuous variables, birthweight, creatinine and eGFR, were nearly normally distributed. Associations of birthweight with outcomes were evaluated using birthweight in sex-specific quintiles, those of LBW vs. normal birthweights, and birthweights as a continuous variable. Parameters of kidney function outcomes were categorized as ‘low’ if they were ≤10th gender-specific percentile and ‘high’ if they were above 90th percentile. Analysis of variance was used to test the difference of the means of eGFR across the birthweight quintiles. In multivariate analyses we adjusted for age, BMI, physical activity, smoking status, alcohol intake, and socioeconomic status (based on education, income and dwelling type). The strength of the relationship between birthweight and dichotomous outcome variables was assessed through logistic regression. We used linear regression to assess the strength of the association between birth weight (per 1 kg increase) and eGFR in females and males separately. For the population attributable risk percentage (PAR%) calculations, those with LBW were regarded as exposed. The PAR% represents the proportion of outcomes in the whole population that might be prevented if all individuals in the population had a birthweight ≥2.5 kg. Stata for windows was used for statistical analyses [27].

The article "Birthweight predicts glomerular filtration rate in adult-life: population based cross sectional study" was retracted in 2022. Reasons: no approval from a third party; copyright claims.

## Results

During the study period, 7157 responded to the administered birthweight questionnaires. About 4502 provided information of their birthweight data. The participants range of birthweight was 0.4–7.0 kg and their birth weight mean (SD) was 3.37 (0.7) kg (Figure 1). The mean (SD) of birthweight was lower for female’s population, of 3.28 (0.6) kg, than males’ population, of 3.5 (0.7) kg. Eight percent (8.0%) had a birthweight less than 2.5 kg. One percent had a birthweight less than 1.5 kg and one percent had a birthweight of five kg and over [28].

**Figure 1.** Shows the birthweight distribution of the participants, which ranged from 0.4 to 7 kg with a mean (SD) of 3.37 (0.7) kg.

As shown in Table 1, people who did not report their birthweight were older and more likely to be female than those who did report their birthweight. They were also shorter and had higher serum creatinine and lower eGFR. Majority (>90%) of participants stated that their birthweight is ‘accurate’ and only six percent mentioned that their birthweight was based on a ‘guess’. Among those who reported their birthweight, 80% obtained their birthweight from a family member, and 10% from medical records. Mean (SD) birthweight was similar for those reported from family members and from medical records 3.35 (0.6) vs. 3.37 (0.7), with adjustment for age and sex, *p* = .36 [28].

**Table 1.** Characteristics of people who provided their birthweight and those who did not provide their birthweight (including both respondents and non-respondents to the birthweight questionnaire).

	with birthweight	without birthweight^a^	
Female			
Numbers	2711	3488	
	Mean (95%CI)	Mean (95%CI)	*p* value
Age, years	48.2 (47.7, 48.8)	53.6 (53.1, 54.1)	<.001
Height, cm	163.2 (163, 164)	161.2 (161,162)	<.001
Weight, kg	70.4 (69.8, 71.0)	70.3 (69.8, 70.9)	.893
Body mass index, kg/m^2^	26.6 (26.4, 26.8)	27.0 (26.8, 27.2)	.005
Albuminuria^b^, mg/l	8.01 (7.72, 8.28)	9.62 (9.30, 9.95)	<.001
ACR^b^, mg/mmol	0.74 (0.72, 0.76)	0.90 (0.87, 0.93)	<.001
Serum creatinine, mg/dl	0.88 (0.88, 0.89)	0.90 (0.89, 0.90)	<.001
eGFR (CG) [22], mls/min	88.0 (87.1, 88.9)	82.6 (81.7, 83.6)	<.001
Male			
Numbers	1791	3257	
	Mean (95%CI)	Mean (95%CI)	*p* value
Age, years	48.3 (47.7, 48.8)	53.6 (53.1, 54.1)	<.001
Height, cm	177.0 (177, 177)	175.0 (175, 175)	<.001
Weight, cm	85.5 (84.9, 86.2)	83.2 (82.7, 83.7)	<.001
Body mass index, kg/m^2^	27.3 (27.1, 27.5)	27.2 (27.1, 27.3)	.496
Albuminuria^b^, mg/l	8.12 (7.79, 8.47)	10.38 (10.01, 10.78)	<.001
ACR^b^, mg/mmol	0.53 (0.51, 0.55)	0.73 (0.70, 0.76)	<.001
Serum creatinine, mg/dl	1.07 (1.06, 1.08)	1.08 (1.08, 1.09)	.022
eGFR (CG) [22], mls/min	103.6 (102, 105)	95.0 (94.0, 96.0)	≤.001

ACR: albumin creatinine ratio; eGFR: estimated glomerular filtration rate; CG: Cockcroft Gaut.

^a^Participants who did not provide their birthweight include (i) those who did not respond to the birthweight questionnaire (*n* = 4090) and (ii) those who answered the questionnaire but could not recall their birthweight (*n* = 2655).

^b^Geometric means.

The article "Birthweight predicts glomerular filtration rate in adult-life: population based cross sectional study" was retracted in 2022. Reasons: no approval from a third party; copyright claims.

Table 2 summarizes the directly measured kidney parameters across birthweight quintiles. People in the lowest birthweight quintile were younger and lighter in weight compared to higher birthweight quintiles. There were trends toward significant differences across birthweight quintiles for albuminuria and albumin-creatinine ratio among females and in males.

**Table 2:** Means (95%CIs) of the direct kidney functions parameters by birthweight quintiles.

Females						
Birthweight, kg	≤2.81	2.81-	3.19-	3.41-	≥3.72	*p* value
Number	546	637	526	466	536	
Age, years	47.1 (46.0, 48.1)	47.8 (46.8, 48.7)	47.2 (46.1, 48.3)	48.7 (47.8, 49.7)	50.6 (49.4, 51.7)	<.001
Weight, kg	69.0 (67.0, 70.2)	69.2 (68.0, 70.4)	70.9 (69.6, 72.1)	71.0 (69.6, 72.3)	73.2 (71.8, 74.6)	<.001
Ualb (gmean)	9.3 (8.5, 10.9)	7.93 (7.38, 8.52)	7.99 (7.38, 8.65)	7.71 (7.09, 8.39)	8.05 (7.45, 8.70)	.050
UCr (gmean)	9.5 (8.03, 10.01)	9.90 (9.46, 10.4)	10.0 (9.51, 10.5)	9.89 (9.38, 10.4)	10.2 (9.71, 10.7)	.058
ACR (gmean)	0.95 (0.80, 0.98)	0.74 (0.69, 0.79)	0.74 (0.68, 0.79)	0.72 (0.67, 0.78)	0.74 (0.69, 0.79)	.033
Serum creatinine	0.89 (0.88, 0.89)	0.88 (0.87, 0.89)	0.86 (0.85, 0.88)	0.87 (0.86, 0.88)	0.89 (0.88, 0.90)	.189
Males						
Birthweight, kg	≤3.06	3.06-	3.37-	3.64-	≥4.05	*p* value
Number	364	355	408	311	353	
Age, years	46.9 (45.6, 48.2)	48.0 (46.8, 49.2)	48.9 (44.4, 50.3)	48.7 (47.4, 50.0)	48.9 (47.8, 50.0)	.177
Weight, kg	82.6 (81.0, 84.2)	81.9 (80.4, 83.4)	85.0 (83.5, 86.5)	86.2 (84.9, 87.6)	89.4 (88.2, 90.7)	<.001
Ualb (gmean)	9.49 (8.74, 10.31)	8.22 (7.53, 8.97)	7.82 (7.12, 8.58)	7.74 (7.02, 8.55)	8.30 (7.56, 9.11)	.050
UCr (gmean)	13.4 (12.7, 14.2)	14.4 (13.7, 15.1)	14.6 (14.0, 15.3)	14.7 (13.9, 16.5)	14.9 (14.2, 15.6)	.093
ACR (gmean)	0.67 (0.63, 0.72)	0.54 (0.50, 0.59)	0.52 (0.48, 0.57)	0.48 (0.44, 0.53)	0.54 (0.50, 0.59)	.044
Serum creatinine	1.09 (1.07, 1.10)	1.07 (1.06, 1.08)	1.06 (1.05, 1.08)	1.07 (1.06, 1.09)	1.07 (1.05, 1.08)	.264

Ualb: albuminuria: mg/L; UCr (gmean) = urinary creatinine: mmol/l; ACR = albumin creatinine ratio, mg/mmol; Serum creatinine = mg/dl; gmean = geometric mean.

The article "Birthweight predicts glomerular filtration rate in adult-life: population based cross sectional study" was retracted in 2022. Reasons: no approval from a third party; copyright claims.

Tables 3 and 4 shows significant differences across birthweight quintiles in eGFR. In females and in males, eGFR were significantly lower in people in the lower birthweight quintiles. This applied to unadjusted and adjusted estimates of eGFR.

**Table 3.** Means (95%CIs) of estimated GFR (ml/min) among birthweight quintiles.

Females						
Birthweight	<2.81	2.81-	3.19-	3.41-	≥3.72	*p* value
CG(22)	85.3 (83.3, 87.4)	87.2 (85.3, 89.2)	88.5 (86.4, 90.6)	88.7 (86.5, 90.9)	90.4 (88.3,92.5)	.008
CG adjusted for age	86.1 (84.5, 87.8)	86.3 (84.6, 88.0)	89.0 (87.1, 90.8)	88.4 (86.4, 88.0)	91.6 (89.5, 93.6)	<.001
CG adjusted for age & BMI	85.9 (84.9, 86.8)	87.4 (86.4, 88.4)	88.7 (87.7, 89.8)	88.6 (87.5, 89.6)	90.6 (89.4, 91.8)	<.001
CG adjusted for age, BMI, alcohol & smoking	85.4 (84.5, 86.4)	87.0 (86.1, 88.0)	88.1 (87.1, 89.2)	88.0 (86.9, 89.1)	90.0 (88.8, 91.2)	<.001
CG adjusted for age, BMI, alcohol, smoking & SES	86.0 (85.0, 86.9)	87.6 (86.6, 88.6)	88.7 (87.6, 89.7)	88.4 (87.3, 89.5)	90.6 (89.4, 91.8)	<.001
CG adjusted for age, alcohol, smoking & SES	85.8 (84.1, 87.4)	86.1 (84.3, 87.8)	88.5 (86.6, 90.3)	87.9 (85.9, 89.8)	90.8 (88.7, 92.9)	.001
CG adjusted for age, diabetes and hypertension	85.1 (83.1, 87.0)	85.2 (83.4, 86.9)	88.4 (86.5, 90.3)	88.9 (86.9, 90.8)	91.7 (89.6, 93.8)	<.001
Males						
Birthweight	<3.06	3.06-	3.37-	3.64-	≥4.05	*p* value
CG(22)	100.3 (97.1, 103)	100.5 (97.9, 103)	101.5 (98.7, 104)	106.6 (104, 109)	110.3 (108, 113)	<.001
CG adjusted for age	100.5 (98.1, 103)	99.5 (97.3, 102)	102.5 (100, 105)	103.9 (102, 106)	108.8 (107, 111)	<.001
CG adjusted for age & BMI	101.5 (99.8, 103)	101.8 (100, 103)	102.5 (101, 104)	104.0 (103, 105)	106.5 (105, 108)	<.001
CG adjusted for age, BMI, alcohol & smoking	100.8 (99.1, 102)	101.2 (99.7, 103)	101.9 (100, 103)	103.6 (102, 105)	105.7 (105, 107)	<.001
CG adjusted for age, BMI, alcohol, smoking & SES	101.3 (99.7, 103)	101.8 (100, 103)	102.5 (101, 104)	104.1 (103, 105)	106.3 (105, 108)	<.001
CG adjusted for age, alcohol, smoking, & SES	100.0 (97.7, 102)	100.9 (100, 103)	102.0 (99.7, 104)	103.2 (101, 105)	107.9 (106, 110)	<.001
CG adjusted for age, diabetes and hypertension	99.7 (97.4, 102.0)	100.4 (98.1, 102.7)	102.5 (100.3, 104.6)	107.2 (104.8, 109.6)	110.0 (107.7, 112.3)	<.001

GFR: glomerular filtration rate; CG: Cockcroft Gault; BMI: body mass index; SES: socioeconomic status based on education, income and dwelling type. Diabetes and hypertension defined according to the World Health Organization definitions.

The article "Birthweight predicts glomerular filtration rate in adult-life: population based cross sectional study" was retracted in 2022. Reasons: no approval from a third party; copyright claims.

**Table 4.** Means (95%CIs) of estimated GFR adjusted for body surface area (ml/min/1.73m^2^) among birthweight quintiles.

Females						
Birthweight	<2.81	2.81-	3.19-	3.41-	≥3.72	*p* value
Number	546	637	526	466	536	
CG(22)	83.0 (81.0, 85.0)	85.5 (83.9, 87.1)	86.0 (84.9, 87.1)	86.7 (85.2, 88.1)	84.0 (81.9, 86.2)	.027
CG adjusted for age	84.4 (82.7, 86.0)	85.2 (83.8, 86.7)	87.3 (85.9, 88.8)	85.9 (84.3, 87.6)	84.7 (83.4,86.1)	.069
CG adjusted for age, alcohol & smoking	84.6 (83.5, 85.7)	85.3 (84.2, 86.4)	86.1 (84.9, 87.3)	85.1 (83.8, 86.3)	86.8 (85.5, 88.2)	.113
CG adjusted for age, alcohol, smoking & SES	84.1 (83.7, 85.3)	84.9 (83.8, 86.0)	86.1 (84.9, 87.3)	85.3 (83.9, 86.5)	86.7 (85.4, 88.1)	.053
Males						
Birthweight	<3.06	3.06-	3.37-	3.64-	≥4.05	*p* value
Number	364	355	408	311	353	
CG(22)	85.8 (83.9, 87.6)	86.2 (84.2, 88.3)	88.5 (86.6, 90.3)	87.4 (85.7, 89.1)	88.8 (87.2, 90.4)	.068
CG adjusted for age	86.3 (84.8, 87.5)	86.9 (85.4, 88.3)	87.0 (85.7, 88.3)	87.2 (86.1, 88.4)	89.3 (88.2, 90.4)	.003
CG adjusted for age alcohol & smoking	86.3 (85.0, 87.6)	86.8 (85.4, 88.2)	87.1 (85.7, 88.4)	87.3 (86.1, 88.5)	89.1 (88.0, 90.2)	.011
CG adjusted for age, alcohol, smoking, & SES	86.3 (85.0, 88.4)	86.9 (85.4, 88.3)	87.1 (85.7, 88.4)	87.2 (86.0, 88.4)	89.1 (88.0, 90.2)	.012

GFR: glomerular filtration rate; CG: Cockcroft Gault; BMI: body mass index; SES: socioeconomic status based on education, income and dwelling type.

**Table 5.** GFR (means, 95%CI), estimated by Cockcroft Gault equation, by birthweight quintiles, stratified by BMI and by age.

Females						
Birthweight	<2.81	2.81-	3.19-	3.41-	≥3.72	*p* value
CG(22), ml/min						
BMI < 25	73.5 (71.5, 75.5)	75.7 (73.9, 77.5)	78.2 (76.3, 80.1)	78.1 (76.0, 80.1)	80.6 (78.6, 82.6)	<.001
BMI ≥ 25	95.8 (92.7, 97.9)	96.7 (93.9, 99.5)	96.3 (93.7, 98.8)	98.0 (95.3, 101)	100 (97.9, 103)	.081
≤ 60 years	89.6 (87.4, 91.8)	91.8 (89.8, 93.8)	92.2 (90.0, 94.3)	92.4 (90.1, 94.7)	96.3 (94.1, 98.6)	<.001
> 60 years	63.0 (60.2, 65.8)	65.4 (62.4, 68.4)	65.8 (62.7, 69.0)	67.1 (64.3, 69.9)	67.7 (64.0, 71.5)	.087
Males						
Birthweight	<3.06	3.06-	3.37-	3.64-	≥4.05	*p* value
CG(22), ml/min						
BMI < 25	90.2 (86.9, 93.6)	88.4 (85.2, 91.7)	92.8 (89.8, 95.9)	95.4 (91.4, 99.3)	93.1 (89.5, 96.6)	.061
BMI ≥ 25	105.0 (102, 108)	106.3 (103, 110)	104.9 (102, 108)	115.1 (112, 119)	111.6 (108, 115)	<.001
≤ 60 years	105.6 (103, 108)	107.5 (105, 110)	106.3 (104, 109)	113.1 (110, 116)	113.1 (110, 116)	<.001
> 60 years	69.8 (65.8, 73.7)	76.8 (72.7, 80.8)	76.9 (73.1, 80.8)	79.6 (75.8, 83.5)	81.1 (74.9, 87.2)	.004

GFR: glomerular filtration rate, ml/min; CG: Cockcroft Gault; BMI: body mass index, kg/m^2^.

The article "Birthweight predicts glomerular filtration rate in adult-life: population based cross sectional study" was retracted in 2022. Reasons: no approval from a third party; copyright claims.

When eGFR formulae were also standardized for 1.73 m^2^ of BSA, the relationships persisted. Due to the smaller BSAs in lower birthweight people, the magnitude of the difference in eGFRs across birthweight quintiles was reduced. Statistical significance was retained amongst males, but was borderline among females, as shown in Tables 3 and 4.

Table 5 shows that the relationships of birthweight with eGFR persisted when participants were stratified by BMI and age categories, though statistical significance was only borderline (*p* = .06–.09) for males with BMI <25 kg/m^2^ and for females with BMI ≥25 kg/m^2^ or aged >60 years.

Table 6 shows the relationship and trends of statistically significant trends by birthweight quintiles in proportions of people with high urine albumin, urine ACR or serum creatinine by birthweight quintile. Point estimates suggest higher rates of elevated urine albumin and ACR in people in the lower birthweight quintiles, but the confidence intervals indicate the differences are not significant in relation to rates of those in the highest birthweight quintiles. However, there were substantially higher proportions with low eGFR levels among females and males in the lowest birthweight quintile. The point estimates for risks for low eGFR in females and males in the lowest birthweight quintiles were 1.35 times and 1.49 times, respectively, compared to those in the highest birthweight quintile, and increased further with adjustment for other factors, to 2.19 and 2.37 times, respectively, which were significant.

**Table 6.** Proportions and odds ratios (OR) and 95%CIs, for high urine albumin, high ACR, high SCr and low GFR by birthweight quintiles.

Females: birthweight, kg		≤2.81	2.81-	3.19-	3.41-	≥3.72	*p* value
Number		546	637	526	466	536	
High ualb	Proportions	0.19 (0.17, 0.21)	0.17 (0.15, 0.19)	0.16 (0.14, 0.190)	0.17 (0.15, 0.91)	0.18 (0.15, 0.19)	.063
	OR^a^ (95%CI)	1.26 (0.97, 1.75)	1.07 (0.72, 1.60)	1.10 (0.73, 1.68)	0.99 (0.64, 1.55)	1.0	
	OR^b^ (95%CI)	1.32 (0.99, 1.73)	1.07 (0.67, 1.69)	0.97 (0.60, 1.58)	0.95 (0.57, 1.56)	1.0	
High ACR	Proportions	0.19 (0.17, 0.21)	0.17 (0.15, 0.20)	0.17 (0.14, 0.20)	0.17 (0.14, 0.21)	0.16 (0.13, 0.19)	.064
	OR^a^ (95%CI)	1.38 (0.98, 1.91)	1.05 (0.70, 1.58)	1.05 (0.69, 1.61)	1.12 (0.78, 1.44)	1.0	
	OR^b^ (95%CI)	1.34 (0.94, 2.14)	1.10 (0.68, 1.77)	1.08 (0.66, 1.76)	1.09 (0.74, 1.58)	1.0	
High SCr	Proportions	0.13 (0.10, 0.15)	0.09 (0.07, 0.12)	0.09 (0.07, 0.12)	0.10 (0.07, 0.13)	0.11 (0.09, 0.14)	.083
	OR^a^ (95%CI)	1.38 (0.97, 1.61)	0.71 (0.49, 1.04)	0.72 (0.48, 1.06)	1.06 (0.71, 1.14)	1.0	
	OR^b^ (95%CI)	1.47 (101, 1.53)	0.84 (0.54, 1.27)	0.80 (0.51, 1.25)	1.08 (0.72, 1.33)	1.0	
Low GFR	Proportions	0.15 (0.12, 0.18)	0.10 (0.08, 0.12)	0.09 (0.07, 0.12)	0.08 (0.07, 0.11)	0.10 (0.07, 0.13)	.044
	OR^a^ (95%CI)	1.35 (0.99, 1.98)	1.15 (0.69, 1.51)	0.94 (0.62, 1.42)	0.94 (0.61, 1.44)	0.10	
	OR^b^ (95%CI)	2.19 (1.14, 4.21)	1.14 (0.58, 2.25)	1.09 (0.81, 2.04))	1.03 (0.54, 1.74	1.0	
Males: birthweight, kg		≤3.06	3.06-	3.37-	3.64-	≥4.05	
Number		364	355	408	311	353	
High ualb	Proportions	0.19 (0.16, 0.22)	0.15 (0.12, 0.19)	0.13 (0.10, 0.17)	0.10 (0.08, 0.14)	0.14 (0.10, 0.18)	.060
	OR^a^ (95%CI)	1.41 (0.95, 1.95)	1.05 (0.65, 1.69)	0.82 (0.49, 1.37)	0.75 (0.44, 1.29)	1.0	
	OR^b^ (95%CI)	1.64 (0.99, 2.89)	1.39 (0.79, 2.43)	0.95 (0.51, 1.77)	0.99 (0.53, 1.87)	1.0	
High ACR	Proportions	0.19 (0.16, 0.22)	0.14 (0.10, 0.17)	0.13 (0.10, 0.17)	0.10 (0.08, 0.14)	0.14 (0.11, 0.18)	.080
	OR^a^ (95%CI)	1.37 (0.97, 1.87)	0.83 (0.50, 1.37)	0.84 (0.51, 1.36)	0.74 (0.43, 1.26)	1.0	
	OR^b^ (95%CI)	1.48 (0.99, 2.46)	1.24 (0.67, 2.30)	0.83 (0.45, 1.56)	0.99 (0.55, 1.77)	1.0	
	High SCr	Proportions	0.13 (0.09, 0.15)	0.08 (0.06, 0.12)	0.09 (0.06, 0.12)	0.07 (0.05, 0.10)	.09 (.07, .13)
	OR^a^ (95%CI)	1.27 (0.95, 1.46)	0.93 (0.56, 1.55)	1.14 (0.71, 1.84)	0.74 (0.42, 1.30)	1.0	
	OR^b^ (95%CI)	1.37 (0.97, 2.28)	1.24 (0.70, 2.19)	1.06 (0.58, 2.07)	1.09 (0.58, 2.07)	1.0	
Low GFR	Proportions	0.13 (0.10, 0.17)	0.12 (0.09, 0.16)	0.11 (0.08, 0.14)	0.04 (0.02, 0.06)	0.10 (0.07, 0.13)	<.001
	OR^a^ (95%CI)	1.49 (0.99, 2.14)	1.38 (0.80, 2.01)	1.23 (0.70, 1.81)	0.34 (0.17, 0.69)	0.10	
	OR^b^ (95%CI)	2.37 (1.06, 5.31)	1.35 (0.64, 2.30)	1.17 (0.74, 1.73)	0.99 (0.35, 2.82)	1.0	

Ualb: Albuminuria: mg/L, high 90th percentile of ualb (females >24.1 mg/l and males >21.6 mg/l); ACR: albumin creatinine ratio, mg/mmol, high 90th percentile of ACR (females >1.95 mg/mmol and males >1.27 mg/mmol); SCr: serum creatinine, high 90th percentile of serum creatinine (females >1.02 mg/dl and males >1.22 mg/dl); GFR: glomerular filtration rate by using Cockcroft Gault equation(22), ml/min, low 10th percentile (females ≤61.4 mL/min and males ≤73.4 mL/min).

^a^Unadjusted.

^b^Adjusted for age, BMI and physical activity (based on time spent on exercise and watching television), smoking status, alcohol intake, and socioeconomic status (2603 of 2711 of females and 1745 of 1791 of males).

The article "Birthweight predicts glomerular filtration rate in adult-life: population based cross sectional study" was retracted in 2022. Reasons: no approval from a third party; copyright claims.

Using the customary definition of low birthweight, < 2.5 kg, which applied in 8.0% of people, (as opposed to the 20% embraced by the lowest birthweight quintile), there were similar differentials in eGFR. Mean eGFR in LBW vs. normal birthweight people was 85.4 (82–88) vs. 88.3 (88–89), *p* = .057, for females and 94.9 (90–100) vs. 104.2 (103–105), *p* < .001 for males. With adjustments for confounding factors, mean eGFR was 85.6 (84.2–87.1) vs. 87.8 (87.3–88.2), *p* = .009 for females, and 94.9 (90–100) vs. 104.2 (103–105), *p* < .001 for males. The mean eGFR/1.73m^2^ was 82.4 (81.2, 84.9) vs. 85.6 (85.2, 85.9), *p* = .048 for females, and 83.2 (80.0, 86.0) vs. 87.8 (87.0, 88.6), *p* = .007 for males. The proportions with low eGFR were 0.14 (0.09–0.18) vs. 0.10 (0.08–0.11), *p* = .053 for females and 0.17 (0.11–0.26) vs. 0.10 ((0.08–0.11), *p* = .015 for males, and the odds ratios (95%CI) for low eGFR, adjusted for other factors were 1.99 (1.08–3.65), *p* = .027, for females and 2.52 (1.63–3.68), *p* < .001 for males.

For each kg increase in birthweight, there was predicted increase in eGFR of 4.5 mL/min (3.5, 5.2), *p* = .043, and75.2 (5.5, 9.0), *p* < .001, for females and males, respectively. The PAR% (95%CI) of LBW for low eGFR was 6.9% (3.5, 11.0) and 7.8% (3.4, 12.6) for females and males, respectively. These values were not significantly changed when adjustments were made for various confounders.

## Discussion

This is the first study to examine the associations of birthweight with eGFR in a well-designed representative of the general Australian population aged over 25 years. There were significant positive relationships, in both females and males, between birthweight and estimated GFR. The association applied when eGFR was expressed in absolute terms, and persisted with adjustment for age, as well as for physical activity, smoking status, alcohol intake and current socioeconomic status. Also, the birthweight was significantly associated with urine albumin levels and with urine albumin:creatinine ratios in this population-based study group.

The findings are consistent with a relationship of birthweight to nephron number, which has now been demonstrated in newborns, children and in adults. Brenner BM and Chertow GM have suggested a direct relationship between birth weight and nephron number [37,38]. Hence, others report compatible with observations that lower birthweight predisposes to the development of chronic kidney disease and its progression, which might be mediated more directly through lower nephron numbers, as inferred here, as well as through higher blood pressures and higher rates of metabolic abnormalities, including dysglycemia and diabetes, to which lower birthweights also predispose.

The article "Birthweight predicts glomerular filtration rate in adult-life: population based cross sectional study" was retracted in 2022. Reasons: no approval from a third party; copyright claims.

The findings support other reports of associations of lower birthweights with kidney disease: A Dutch study, of 422 (46.7% males) participants with a mean (SD) age of 19.3 (0.2) years, found that intrauterine growth retarded subjects born very premature were at increased risk of developing kidney disease in later life [29]. Furthermore, In the United States, Lackland et al. reported a U-shaped quadratic association between birthweight and early onset kidney disease in participants living in the southeast of USA [30]. However, the majority were non-Caucasians. In Canada, women from the Saskatchewan population with ESKD were three times more likely to have had LBW compared with subjects without ESKD [31]. Lackland et al. found that ESKD [32,33] and the odds of chronic kidney disease by low birthweight was highest in patients with both diabetes and hypertension [30,34]. We found that urban Australian patients with chronic kidney disease (CKD) had lower birth weights than their matched Australian controls. In addition, the more advanced the CKD stage, the lower the birth weight [35].

In recent years, there has been great interest in the early development of the fetus and the impact of growth during the gestational period on the development of diseases in later life, and that termed a ‘critical period’ [36]. The ‘critical period’ of growth of various tissues and organs is the rapid growth period that starts from the ninth week of gestation onwards, which is determined by rapid cell division. Disproportionate development of various structures and or different organ systems in pre-natal life can occur because different tissues have different critical periods of growth at different times of development *in utero* [37,38].

There are many reports that LBW, < 2.5 kg, predisposes to many diseases including hypertension, diabetes, cardiovascular diseases, and kidney diseases. However, most previous studies found a significant relationship when adjustments were made for body mass index (BMI) or current body weight. Also, many studies were criticized for not adjusting for important confounders such as physical activity, smoking status, alcohol intake, family history and socioeconomic factors [16,17,39,40].

In the Australian population, where general health is good and most birthweights are within normal range, the impact of lower birthweights on population-based rates of kidney disease is probably not great, as indicated by the modest population attributable fractions for low eGFR associated with birthweights < 2.5 kg. The phenomenon does, however, flag potential increase in risk for chronic kidney disease and the attendant end-stage kidney disease risk in lower birthweight people, and perhaps the advisability of heightened surveillance. From a global health perspective but more in developing countries and in populations in epidemiologic transition, where substantially lower birthweights coexist with recently improved infant and adult survivals, the overall impact of this phenomenon on the population health profile could be more substantial.

The article "Birthweight predicts glomerular filtration rate in adult-life: population based cross sectional study" was retracted in 2022. Reasons: no approval from a third party; copyright claims.

This phenomenon, of low birthweight contributing to later development of chronic diseases, has added consequences for the kidney disorders in every country where the prevalence and incidence of low birthweights is increasing, and the newborns survive. The improvement in intensive care and other various medical care with time have permitted those with lower birthweight infants to endure better survival to adult life. Worldwide, in all populations, a secular movement toward higher levels of body fat and BMI have possibly complexes the potentiation of other risk factors such as glycemic abnormalities expression associated with lower birthweights. Modest increases in body fat might have a trivial impact on metabolic and renal diseases burden when acting in isolation, but substantial impact when other risk factors are also operating. It would be pragmatic, to implement strategies of intensified whole of life surveillance of lower birthweight people, foreseeing this risk. Also, in more developed countries, LBW, as the earliest known risk factor, would add a value to the risk stratification for early identification of kidney disease or its various parameters and risk factors [41]. This may guide the point of care decision for further testing and management selection that sets a platform for risk reduction based on biological platform stratification [41].

The role of small size at birth with low number of cells may contribute to various NCD problem [2–5,42–46]. Post-natal environmental factors further compound such a metabolic demand on body organs that lead to various organ function being overwhelmed with increase in metabolic rate. Hence, this primes to upsurge demand upon many human organs or structures, such as pancreatic cells or nephron with subsequent hyperfiltration, and therefore organ dysfunction ensues. Hence, an early tactic health approach and maintenance of comprehensive health-program is of great importance to be instituted to detect major risk factors which may arise early in life in those population of LBW and or prematurity, which is progressively rising world-wide. The logistic and financial requirement may not be huge to put such a strategy forward, but this strategy would in long term delay or even ameliorate the progressive rise of NCD. Hence, endorsing healthier lifestyles, body weight, blood pressure and enhancing the family physicians’ capability should be required to reduce the burden of NCDs. Findings of various risk factors at early post-natal life, such as proteinuria and treatment with angiotensin converting enzyme inhibitors, will help to better manage this subset of our population that is increasing progressively with advancement of medical care for small babies.

The article "Birthweight predicts glomerular filtration rate in adult-life: population based cross sectional study" was retracted in 2022. Reasons: no approval from a third party; copyright claims.

Clinical and experimental data suggest that an inappropriate intrauterine environment may permanently modify the structure of the kidney. This is evidenced not only by reduced nephron number, but also by a compensatory maladaptive change that occurs intra renal when nephrogenesis is compromised. It must be recognized that the high risk for kidney disease associated with fetal programming could be a direct consequence of impaired nephrogenesis or a cumulative process superimposed on type 2 diabetes and the various cardiovascular diseases risk factors [47].

The correlation between glomerulogenesis, glomerular number and glomerular filtration rate is very much intertwined. Although immaturity is associated with impaired nephrogenesis, Faa et al. showed that kidney maturation continues after birth, and that nephrogenesis is a process not restricted to the intrauterine life but is an ongoing process for a period of a few weeks after delivery [48]. Also, postnatal active glomerulogenesis is not restricted to preterm infants, but it may be present in term infants with birthweight in the normal range. This variation in nephron number demonstrates the plasticity of the developing kidney, and the significant role one’s environment plays in determining one’s final nephron count. A marked interindividual variability exists even in preterm infants with the same gestational age at birth. These variabilities possibly due to various stressors which might impair nephron formation during gestation and in the perinatal period [48].

As a new concept of primary prevention of renal disease, Faa et al. suggested that it should start in the perinatal period aimed at increasing the number of functioning glomeruli [49]. This physiological regenerative medicine includes endogenous renal stem cells and stem cell stimulators physiologically expressed in human cells. The renal stem cells in the perinatal period, might transform preterm babies from susceptible to resistant subjects to CKD later in life, in childhood or in adulthood [49].

The article "Birthweight predicts glomerular filtration rate in adult-life: population based cross sectional study" was retracted in 2022. Reasons: no approval from a third party; copyright claims.

The main goal of a regenerative medicine in the perinatal period is to allow preterms and all low-birth-weight infants to reach a sufficient nephron number, protecting their nephrogenesis till its physiological end around the 38th week of postconceptional life [50]. Hence, this enables the transformation of oligonephronic subjects susceptible to develop kidney disease in adulthood, into normonephronic subjects, preventing the insurgence of renal disease later in life [50].

As it is well known for long period, the average number of nephrons per kidney is approximately 1,000,000, but there is a significant amount of variation within the human population. Fanni et al. argue that more attention should be focused on defining, evaluating, and promoting the factors stimulating mitosis and nephrogenesis and inhibiting apoptosis [51]. They suggest defining this approach to a possible therapy of a deficient nephrogenesis at birth calling it the physiological renal regenerating medicine. They argue for the prolongation of the nephrogenesis not only for 6 weeks after birth but until 36 weeks of post conceptual age, allowing newborn kidneys to restore their nephron endowment, escaping susceptibility to hypertension and to renal disease later in life [51]. Although they suggest to program the increase of nephron number during the first few weeks of postnatal life, however intervention trials are needed to evaluate the impact of changing a combination of pre- and post-natal factors on renal health of newborns and children.

Further follow up of this cohort over the coming few years will provide even better data regarding the effect of birthweight on the development of chronic kidney disease and other chronic diseases. In addition, it will provide information on the role of birthweight in the progression of chronic diseases, such as chronic kidney disease, that would add a valuable contribution and strengthen our understanding of the role of fetal development on chronic diseases in adult life. The LBW population is increasingly surviving into adulthood and their risk factor for development of chronic disease should be monitor early, taking into consideration their prenatal and postnatal environmental risk factors that set the cycle of health deterioration.

Primary prevention strategy should be directed toward improvement of maternal health as the utmost important public health concern to ameliorate the LBW as far as possible with empowerment of women and provision of full support. If primary prevention was not successful, then secondary prevention strategy entails close monitoring of those born with LBW and comprehensive management strategy with at least yearly clinical checkup and possible simple laboratory tests such as urinalysis. These simple steps will have a long-lasting cost effective and alleviate burden of non-communicable disease in the populations world-wide.

The article "Birthweight predicts glomerular filtration rate in adult-life: population based cross sectional study" was retracted in 2022. Reasons: no approval from a third party; copyright claims.

Limitations: The analysis of the present study is limited by not including the gestational age. This limits analysis by small for gestational age, appropriate for gestational age and large for gestational age comparison of the population. Also, the study was conducted among Australian people and the study used a self-recall questionnaire to obtain birthweight data. We opted for this method of obtaining birthweight as there are no readily available data banks pf birthweights that cover the AusDiab study population. Many seminal studies, which have reported associations of birthweight with adult health, have employed this technique [52–55], with response rates often less than described here. The British Telecom study had a 50% response rate and only 39.4% provided data on birthweight [53], the British Women’s Heart and Health Study had a 60% response rate and 33% reported their birthweight [54] and the Health Professional Follow-up Study (HPFS) had a 75% response rate and 59% of the responders reported their birthweight [52].

Among birthweight respondents, it is reassuring that the mean birthweight of those who guessed their birthweight; 3.34 (0.6) was like those who obtained their birthweight from a family member; 3.37 (0.6), or from medical records; 3.35 (0.7), *p* = .46. This was also the case in the British Telecom Study [53]. In addition, the mean recalled birthweight in our study, 3.37 (0.7) kg, is consistent with that reported in the United Kingdom in those born between 1931 and 1939 in Hertfordshire [56]; with the 1946 national birth cohort [57]; with the Health Professional Follow Up Study [52] and is similar to the recent average Australian birthweight of 3.36 kg [58].

## Conclusions

Birthweight had a positive relationship with eGFR. Possible explanations include an association of birthweight with nephron-endowment. From a global health perspective but more in developing countries and in populations in epidemiologic transition, where substantially lower birthweights coexist with recently improved infant and adult survivals, the overall impact of this phenomenon on the population health profile could be more substantial.

## Data Availability

Data of this paper is part of the AusDiab study and not available publicly but information available at https://www.baker.edu.au/ausdiab/

## Appendix

### Methods

All subjects attended a local screening venue and completed a series of questionnaires, physical examinations, and specific laboratory tests which examined diabetic status, cardiovascular risk factors, and kidney function. An interviewer-administered questionnaire was used to determine smoking status, alcohol consumption, leisure-time physical activity and television viewing. Assessment of socioeconomic status was based on education, dwelling type and income.

The article "Birthweight predicts glomerular filtration rate in adult-life: population based cross sectional study" was retracted in 2022. Reasons: no approval from a third party; copyright claims.

Participants self-reported their frequency and duration of physical activity during the previous week. Physical activity was measured by the Active Australia questionnaire, which asks respondents about their participation in predominantly leisure-time physical activities (including walking for transport) (30). These questions have been found to provide reliable and valid estimates of adult physical activity (30). Total physical activity time was calculated as the sum of the time spent walking (if continuous and for ≥10 min) or performing moderate-intensity physical activity, plus double the time spent in vigorous-intensity physical activity (31). Frequency of physical activity was calculated by summing the number of sessions of vigorous activity, moderate activity, and walking. Physical activity was categorized to reflect the current Australian public health recommendation for physical activity (31) as active (≥150 min/week across at least five sessions) and inactive (<150 min/week and/or fewer than five sessions).

Participants also self-reported the total time they spent watching TV or videos in the previous week. This measure provides a reliable and valid estimate of TV time among adults (32). The average hours watching TV per week were used to create three categories of TV viewing (0–7, 7.01–14, and > 14 h/week).

During the 2004–2005 follow-up AusDiab survey, questions about birthweight were included. Participants were asked to state their birthweight, the likely accuracy of the stated birthweight and the source of their stated birthweight. Birthweights were recorded as pounds and ounces or in kilograms (kg) and grams. All values were converted to kilograms for analyses. Low birth weight (LBW) is defined by the World Health organization (WHO) as a birth weight of an infant of 2499 g or less (<2.5 kg) (33). Participants were also divided into birthweight quintiles (about 900 participants in each group).

At baseline, all participants except those who were (i) chairbound, (ii) pregnant or (iii) too unsteady on their feet underwent anthropometric measurements while wearing light clothing and no footwear. The methods have been previously described. Briefly, height was measured to the nearest 0.5 cm using a stadiometer, and weight was measured using a mechanical beam balance, and was recorded to the nearest 0.1 kg. BMI was calculated as weight (kg)/height (m)^2^. BMI was defined as < 25 kg/m^2^ and ≥ 25 kg/m^2^ according to World Health Organization criteria (36).

The article "Birthweight predicts glomerular filtration rate in adult-life: population based cross sectional study" was retracted in 2022. Reasons: no approval from a third party; copyright claims.

Blood was collected by venepuncture after an overnight fast of at least 10 h. Blood specimens collected were centrifuged on-site and transported daily with urine samples to the central laboratory. SCr was measured by the modified kinetic Jaffe reaction using the Olympus AU600 auto-analyzer and the coefficient of variation was <1.9%. Urinary albumin and creatinine levels were determined in a spot morning urine specimen by means of enzymatic methods (Olympus AU600 analyzer).

The estimated GFR was obtained using both the MDRD (Modification of Diet in Renal Disease) Study equation (37) and CKD-EPI (Chronic Kidney Disease Epidemiology Collaboration) equation (38), as shown below. Although indexing GFR to body surface area (BSA) is controversial (41), we also describe GFR estimates adjusted for BSA, using the formula: weight (0.425) × height (0.725) × 0.20247 m^2^.

The estimated glomerular filtration rate (eGFR) Equations.

**Table:**

CKD-EPI	
Female; SCr ≤ 0.7 mg/dl	144 × (SCr/0.7)^−0.329^ × 0.993^Age^ [×1.159 if black]
Female; SCr > 0.7 mg/dl	144 × (SCr/0.7)^−1.209^ × 0.993^Age^ [×1.159 if black]
Male; SCr ≤ 0.9 mg/dl	141 × (SCr/0.9)^−0.411^ × 0.993^Age^ [×1.159 if black]
Male; SCr > 0.9 mg/dl	141 × (SCr/0.9)^−1.209^ × 0.993^Age^ [×1.159 if black]
MDRD equation	
	186×(SCr mg/dl)-1.154 × (age)^−0203^ ×0.702 [if Female] × 1.212[if Black]

MDRD: Modification of Diet in Renal Disease; CKD-EPI: Chronic Kidney Disease Epidemiology Collaboration; SCr: serum creatinine.

#### Statistical analysis

Albuminuria, urinary creatinine and ACR were not normally distributed and were logarithmically transformed. The other continuous variables, birthweight, creatinine and eGFR, were nearly normally distributed. Associations of birthweight with outcomes were evaluated using birthweight quintiles, those of LBW vs. normal birthweights, and birthweights as a continuous variable. Parameters of kidney function outcomes were categorized as ‘low’ if they were ≤ 10th percentile and ‘high’ if they were above 90th percentile. Analysis of variance was used to test the difference of the means of eGFR across the birthweight quintiles. In multivariate analyses we adjusted for physical activity, smoking status, alcohol intake, and socioeconomic status (based on education, income, and dwelling type). The strength of the relationship between birthweight and dichotomous outcome variables was assessed through logistic regression. We used linear regression to assess the strength of the association between birth weight (per 1 kg increase) and eGFR.
